# Anterior Bone Loss after Cervical Baguera C Disc versus Bryan Disc Arthroplasty

**DOI:** 10.1155/2023/8010223

**Published:** 2023-02-06

**Authors:** Chih-Chang Yang, Tse-Yu Chen, Wen-Hsien Chen, Chung-Yuh Tzeng, Chih-Wei Huang, Ruei-Hong Lin, Ting-Hsien Kao, Hsien-Te Chen, Chien-Chun Chang, Hsi-Kai Tsou

**Affiliations:** ^1^Department of Neurosurgery, Neurological Institute, Taichung Veterans General Hospital, Taichung, Taiwan; ^2^Division of Neurosurgery, Department of Surgery, Puli Branch, Taichung Veterans General Hospital, Puli Township, Nantou County, Taiwan; ^3^Ph.D. Program in Translational Medicine, National Chung Hsing University, Taichung, Taiwan; ^4^Rong Hsing Research Center For Translational Medicine, National Chung Hsing University, Taichung, Taiwan; ^5^Department of Radiology, Taichung Veterans General Hospital, Taichung, Taiwan; ^6^Department of Industrial Engineering and Enterprise Information, Tunghai University, Taichung, Taiwan; ^7^Department of Orthopedics, Taichung Veterans General Hospital, Taichung, Taiwan; ^8^Department of Medicinal Botanicals and Health Applications, Da-Yeh University, Changhua County, Taiwan; ^9^Institute of Biomedical Sciences, National Chung Hsing University, Taichung, Taiwan; ^10^Functional Neurosurgery Division, Neurological Institute, Taichung Veterans General Hospital, Taichung, Taiwan; ^11^Department of Sports Medicine, College of Health Care, China Medical University, Taichung, Taiwan; ^12^Department of Orthopedic Surgery, China Medical University Hospital, Taichung, Taiwan; ^13^Spine Center, China Medical University Hospital, Taichung, Taiwan; ^14^Department of Rehabilitation, Jen-Teh Junior College of Medicine, Nursing and Management, Houlong, Miaoli County, Taiwan; ^15^Department of Post-Baccalaureate Medicine, College of Medicine, National Chung Hsing University, Taichung, Taiwan; ^16^College of Health, National Taichung University of Science and Technology, Taichung, Taiwan

## Abstract

**Objectives:**

The objectives of this study were to identify the risk factors and incidence of anterior bone loss (ABL) after Baguera C cervical disc arthroplasty (CDA) and identify whether design differences in artificial discs affect ABL.

**Methods:**

In this retrospective radiological review of patients who underwent single-level Baguera C CDA in a medical center, the extent of ABL and the following radiological parameters were recorded: global and segmental alignment angle, lordotic angle (or functional spinal unit angle), shell angle, global range of motion (ROM), and ROM of the index level. ABL at the index level was grade 0-2. Grade 0 was defined as no remodeling, grade 1 as spur disappearance or mild change in body contour, and grade 2 as obvious bone regression with Baguera C Disc exposure.

**Results:**

Combining grade 1 and grade 2, ABL was found in 56 upper adjacent vertebrae and 52 lower adjacent vertebrae of the 77 patients. Only 18 patients (23.4%) had no ABL. Shell angle differed significantly between ABL grades of both the upper and lower adjacent level: 0.0° in grade 0 and 1 ABL vs. 2.0° in grade 2 ABL of the upper adjacent level (*p* < 0.05); and 0.0° in grade 0 and 1 ABL vs. 3.5° in grade 2 ABL of the lower adjacent level (*p* < 0.05). A female predominance of ABL was found. Hybrid surgery and artificial disc size were also related to ABL.

**Conclusions:**

ABL is more common in Baguera C Disc arthroplasty than Bryan Disc arthroplasty. Larger shell angle was related to ABL after CDA with Baguera C Discs, which may indicate that shell angle is pivotal in determining the incidence of ABL after CDA. Females had more ABL with Baguera C Disc arthroplasty; this might be related to shorter endplate lengths as well as a smaller endplate-implant mismatch.

## 1. Introduction

The well-established anterior cervical discectomy and fusion surgical procedure is commonly used for cervical spondylosis. Since its introduction in the 1950s by Smith and Robinson [1] and also Cloward [2], excellent clinical results have been reported in the treatment of degenerative disorders of the cervical spine with radiculopathy or myelopathy. The main disadvantage is that this procedure turns a functional cervical spinal unit into a nonfunctional unit.

Cervical arthroplasty with artificial disc was developed to maintain the mobility of a functional spinal unit. Cervical disc arthroplasty (CDA) was first published in the medical literature by Reitz and Joubert [3] in the South African Medical Journal in 1964. Since then, the cervical disc prosthesis design has been modified based on clinical results and advancements in material science. Despite improvements in technique as well as implant designs in CDA, complications—including metallosis [4], heterotopic ossification (HO) [5], hypermobility, subsidence [6–8], and prosthesis migration [6–8]—still remain.

Anterior bone loss (ABL) in CDA has been reported with both the Bryan Disc [9, 10] and the Baguera C Disc implants [11]. The reported risk factors for severe ABL include greater use of cauterization during surgery, disruption of the anterior longitudinal ligament, less abundant blood supply, and detachment of the collis longus muscle, which may subsequently lead to excessive micromotion [9]. Kim et al. [10] reported bone loss immediately posterior to the Bryan Disc flange. At the early follow-up time points, three patients had bone loss immediately posterior to the anterior Bryan Disc flange on the superior adjacent vertebra. Heo et al. [11] described ABL as a potential complication after CDA, reporting bone loss at the operative segments in 29 (60.4%) of 48 patients treated with Baguera C Disc. Kieser et al. [12] reported ABL in 63.7% of CDAs: 56 with Bryan, 44 with Discocerv, 37 with Mobi-C, and 56 with Baguera C devices. In that study, association with ABL was most significant with Mobi-C compared to Bryan, Discocerv, or Baguera C. These researchers found no significant relationship between the degree of ABL and patient pain at 3 months. Wu et al. [13] found that 224 (56.6%) of 396 patients had ABL at the arthroplasty level when the Prestige-LP Disc was used. Another study reported a greater than expected number of patients with ABL after CDA with Bryan Discs (68 of 121 patients), suggesting that the incidence of ABL after CDA may increase with increasing shell angle. The authors proposed that ABL is a result of increased bone remodeling due to uneven load force distribution and excessive micromotion during the osteointegration process [9].

Our hypothesis is that the shell angle affects the rate of ABL after CDA with both flanged (Bryan) and nonflanged (Baguera C) artificial discs, because the impact of the shell angle on the distribution of the loading force leads to bone remodeling in both implant types. This study is therefore aimed at determining the incidence and risk factors related to ABL after Baguera C CDA and identifying whether design differences between the Baguera C Disc (Spineart, Geneva, Switzerland) and Bryan Disc (Medtronic Sofamor Danek, Memphis, TN, USA) affect the extent of ABL after arthroplasty.

## 2. Methods

### 2.1. Study Population

We conducted a retrospective analysis of patients who underwent single-level Baguera C CDA between August 2014 and July 2020 at a regional center for spine surgery. The surgical indications for CDA included single-level or multilevel disc herniation at C3 to C7 with radiculopathy, myelopathy, or both, with minimal spondylosis. We did not perform CDA in patients with instability, deformity, osteoporosis, metabolic bone disease, or history of cervical spine infection. We reviewed the records of a total of 205 patients treated by the same neurosurgeon to reduce surgeon-related factors. Cases with CDA at more than one level (125 patients) were excluded. However, in order to examine whether fusion in the adjacent segment was a risk factor for ABL, hybrid cases were not excluded. Three patients were excluded because the follow-up period after CDA was less than 12 months. A total of 77 patients were included in the analysis. This study was conducted in accordance with the Declaration of Helsinki (1964) and approved by the institutional ethics committee (CG21045A), which waived the requirement for informed consent.

### 2.2. Radiological Parameters

Comparative radiological measurements were collected before and at 6 months after the operation. Extent of ABL was evaluated at 1, 3, 6, 12, and 24 months postoperation. We calculated the global and segmental alignment angle, shell angle, and lordotic angle (or functional spinal unit [FSU] angle). Radiological parameters were based on lateral radiographs taken when the patient was in a relaxed, neutral position (Figure 1(a)). The measurements were evaluated by two senior and experienced neurosurgeons and were confirmed by an independent neuroradiologist. The global alignment angle was determined using the Harrison posterior tangent method of measuring the angle formed by a line projected parallel to the posterior surface at C2 and a line parallel to the posterior surface at C7 [14]. The segmental alignment angle was defined by the vertebral body tangents of the surgical level, similar to the Harrison tangent method. The lordotic angle was the angle between the upper endplate of the cranial-adjacent level of the implant and the lower endplate of the caudal-adjacent level. The shell angle was defined as the angle formed between the two titanium endplates of the Baguera C Disc. Global and segmental range of motion (ROM) were calculated as described [9]; briefly, these are the differences in the alignment angle between the flexion and extension positions (Figures 1(b) and 1(c)). The anteroposterior diameter of the endplates and implants were measured on a neutral lateral radiogram immediately postoperation. The actual implant depth served as an internal calibration reference [15]. The adjusted anteroposterior diameter of the endplate was calculated using the following equation:x

(1) $$\begin{array}{c} \text{measured diameter of the endplate}\times \frac{\text{actual depth of the implant}}{\text{measured depth of the implant}}. \end{array}$$

The mismatch between the endplate and the implant was calculated as follows:

(2) $$\begin{array}{c} \text{adjusted anteroposterior diameter of the endplate}–\text{actual implant depth}. \end{array}$$

The preoperative disc height of the index level was measured at the anterior aspect, the midpoint, and the posterior aspect of the preoperation neutral lateral radiogram and adjusted according to the following equation:

(3) $$\begin{array}{c} \text{measured diameter of the disc height}\times \frac{\text{adjusted anteroposterior diameter of the endplate}}{\text{measured anteroposterior diameter of the endplate }}. \end{array}$$

The mean disc height was then calculated:

(4) $$\begin{array}{c} \frac{\text{adjusted disc height of anterior aspect}+\text{adjusted disc height of midpoint}+\text{adjusted disc height of posterior aspect}}{3} \end{array}$$

A graded classification of ABL in the operative segments was done as follows (Figure 2). ABL was graded from 0 to 2. Grade 0 was defined as having no remodeling, grade 1 was defined as having spur disappearance (1a) or mild change in body contour (1b), and grade 2 was defined as having obvious bone regression with Baguera C Disc exposure. In grade 1 ABL, we did not differentiate spur disappearance from mild body contour change. These two phenomena often coincide, and the changes are subtle, making them difficult to distinguish from one another. Some examples are shown in Figure 3.

### 2.3. Statistical Analysis

Continuous variables were expressed as median (1^st^ quartile, 3^rd^ quartile). Categorical variables were expressed as count and percentage. Comparisons to determine statistical significance were performed using the Mann−Whitney *U*-test for continuous variables and the chi-square test for categorical variables. The results were considered significant for *p* values < 0.05. Analyses were performed using the Statistical Package for the Social Sciences, version 22.0 (IBM Corp., Armonk, NY, USA).

## 3. Results

A total of 77 patients (40 females and 37 males) were included, and the mean age was 55.9 years. The posterior longitudinal ligament and posterior uncinate processes were resected in all patients. The majority of operative segments were at the C5-C6 (37 cases) and C4-C5 (20 cases) levels, followed by the C3-C4 (17 cases) and C6-C7 (3 cases) levels. Overall, 38 patients underwent 1-level CDA, and 39 patients had a hybrid procedure with concomitant fusion at the same time as CDA. The detailed demographic data for these cases is summarized in Table 1.

Grade 1 upper adjacent vertebra ABL was present in 36 patients (46.8%) and grade 1 lower adjacent vertebra ABL was present in 40 patients (51.9%). Twenty patients (26.0%) had grade 2 upper adjacent vertebra ABL and 12 patients (15.6%) had grade 2 lower adjacent vertebra ABL. Among the 77 patients, there was a total of 56 upper adjacent vertebrae ABL (grade 1 and grade 2) and 52 lower adjacent vertebrae ABL (grade 1 and grade 2). Only 18 patients (23.4%) had no ABL at all. With this high incidence of ABL, the statistical analysis between those with and those without ABL (grade 0 versus grades 1 and 2) yielded nothing notable. Therefore, we present analysis of those with no or minor change (grade 0 and grade 1) versus those with prominent body contour change with artificial disc exposure (grade 2).

ABL was identified one month after the operation, with progression during the first year, mostly occurred 6 to 12 months after the operation, and rarely progressed beyond a year, regardless of the location of the adjacent vertebra (Figures 4(a) and 4(b)). Grade 2 ABL caused anterior artificial disc uncovering, but no significant implant subsidence was noted. In addition, no severe HO or autofusion was observed in patients with ABL.

Similar to reports from the literature, our study found that age and operative level had no effect on ABL. However, we found that ABL was more prevalent in females (85% and 83.3% of cases with grade 2 ABL in the upper and lower adjacent vertebra, respectively, were female patients, *p* < 0.05, Tables 2 and 3).

Hybrid surgery and artificial disc height were related to ABL. CDA was associated with a higher incidence rate of grade 2 ABL, compared to hybrid surgery involving concomitant fusion (75.0% and 83.3% of cases with grade 2 ABL in the upper and lower adjacent vertebra, respectively, underwent CDA only, *p* < 0.05, Tables 2 and 3). Cases with smaller artificial disc heights were also prone to grade 2 ABL (*p* < 0.01, Tables 2 and 3). In addition, smaller artificial disc depths were related to grade 2 ABL of the upper (Table 2), but not the lower, adjacent level (Table 3). Another parameter correlated with artificial disc height, the preoperative disc height, was also significantly smaller in those with grade 2 ABL of the upper adjacent level, but showed only a nonsignificant trend in grade 2 ABL of the lower adjacent level (Tables 2 and 3).

Similar to a previous study on Bryan Discs [9], which reported the effect of shell angle on the extent of ABL, we found a significant difference in shell angle between ABL grades in both the upper and lower adjacent levels. These were 0.0° in grade 0 and grade 1 ABL vs. 2.0° in grade 2 ABL of the upper adjacent level (*p* < 0.05) (Table 2) and 0.0° in grade 0 and grade 1 ABL vs. 3.5° in grade 2 ABL of the lower adjacent level (*p* < 0.05) (Table 3). No correlation to ABL was found for the other radiological parameters, including global alignment angle, lordotic angle (FSU angle), or global and index level ROM.

Female patients tended to have smaller endplates and smaller artificial discs (both in height and depth) used during CDA. The adjusted diameter as well as the endplate-implant mismatch were smaller in female patients than in male patients (*p* < 0.01, Table 4). As a result, interactions might exist between female sex, the depth/height of the implant, the endplate diameter, and the endplate-implant mismatch.

## 4. Discussion

### 4.1. Shell Angles Were Strongly Related to ABL in CDA with Both Bryan and Baguera C Discs

Our results showed that larger shell angles were related to ABL after CDA with Baguera C Discs. These results were consistent with a similar study on ABL with Bryan Discs [9]. Shell angle very likely plays a pivotal role in predicting the incidence of ABL after CDA. To our surprise, our patients who underwent arthroplasty with Baguera C Disc had a higher rate of ABL than that reported in previous studies [11, 12, 16].

### 4.2. Female Predominance Was Found in ABL with Baguera C Discs

In addition, a female predominance existed in ABL after CDA with Baguera C Discs. There was no sex difference in those receiving Bryan Disc arthroplasty and the exact mechanism remains unclear. Most likely, this difference reflects an interaction between various factors attributable to hormone-related physiology. We did identify that female patients tended to have smaller adjusted anteroposterior diameter and smaller endplate-implant mismatch (Table 4), both of which were significantly related to ABL (discussed below).

The smaller height of Baguera C Discs was also associated with a greater incidence of ABL. Theoretically, the height of artificial discs should be related to the preoperative disc height, because only smaller implants would fit into the smaller disc spaces. In fact, smaller preoperative disc height was associated only with ABL in the upper adjacent vertebra, with no association found in the lower adjacent vertebra. The exact mechanism of the correlation remains to be elucidated in future studies.

### 4.3. Endplate-Implant Mismatch Plays a Crucial Role in Bone Remodeling

In our study, we found that a smaller mismatch between the endplate and the artificial disc was associated with a greater likelihood of ABL (Tables 2 and 3). On the other hand, in studies of the uncovered endplate, or the residual exposed endplate (REE) value [17], larger REE was associated with anterior HO after CDA [18, 19]. These findings suggest the intriguing idea that the mismatch between the endplate and the artificial disc (or footprint mismatch) plays a major role in postoperative bone homeostasis: a smaller mismatch would tilt the equilibrium of bone remodeling towards bone resorption, and a larger mismatch, or larger REE, would favor bone formation leading to HO. In a recent study by Wang et al. of 70 patients who underwent 1-level CDA with Prestige-LP, the authors concluded that ABL might be the opposite of anterior HO [20]. They also found that patients with anterior HO had a kyphotic disc angle after surgery, while patients with ABL had a lordotic disc angle after surgery. These results are consistent with our finding that larger shell angle (disc angle) was associated with a greater incidence of ABL.

### 4.4. Bryan versus Baguera C Discs

Several aspects of the design, structure, surgical procedure, and postoperative biomechanics account for the differences between Bryan and Baguera C Discs.

First, focal segmental kyphosis with preserved global alignment and segmental motion have all been reported after Bryan Disc arthroplasty [7, 21–24]. It is postulated that asymmetrical endplate milling and intraoperative lordotic distraction are the main reasons for postoperative segmental kyphosis [23]. Such segmental kyphosis after Bryan Disc arthroplasty implies a smaller shell angle compared with the normal lordotic shell angle after Baguera C Disc arthroplasty which, as theorized [9], would lead to a lower incidence of ABL due to uneven force distribution.

Second, the Baguera C Discs are placed deeper into the disc space, with no flange as in Bryan Discs. Bryan Discs have perpendicular, punched flanges (anterior stop), bent cephalad on the upper shell and caudal on the lower endplate [24], which prevent posterior displacement of the device into the spinal canal. On the other hand, Baguera C Discs are placed deeper, with the posterior aspect of the shells parallel to the posterior aspect of the vertebral bodies, thus placing them closer to the center of gravity (Figures 5 and 6). The difference in depth of placement between Bryan Discs and Baguera C Discs may lead to a different distribution pattern of the loading force. The smaller loading force at the anterior aspect of the cervical vertebrae after CDA with Baguera C Discs may have contributed to the increased incidence of ABL.

Third, the anterior cervical osteophytes were removed during the endplate preparation process in CDA with Bryan Discs [23]. However, we did not need to resect the anterior cervical osteophytes in CDA with the Baguera C Discs. As a result, while resorption of anterior marginal spurs after Baguera C Discs was considered as grade 1a ABL, the same resorption of anterior marginal spurs was masked with Bryan Discs, due to spur removal during surgical procedure. In fact, the incidence of ABL with Baguera C Discs may more closely reflect the true prevalence of bone remodeling after CDA.

Lastly, the Baguera C Disc is a semiconstrained device with a mobile-core mechanical property and a shock-absorbing function. In addition, no liftoff phenomenon, spontaneous movement during the loading condition, or significantly lower contact pressure distribution on the core was observed, which can be interpreted as a lower likelihood of long-term wear inside the core [25]. Theoretically, the Baguera C Disc has less harbor dust than the Bryan Disc from the burring and milling procedure. However, our data showed more ABL in Baguera C Discs. These phenomena serve as another strong argument against regarding ABL as merely an interaction between wear debris and osteolysis.

### 4.5. Osteolysis Is a Different Phenomenon

In a recent review article, the authors cited the same classification of ABL as used here and concluded that ABL following CDA is mostly not due to remodeling [26]. The cited study [9] clearly stated that ABL was a remodeling process. ABL and osteolysis are two different phenomena with distinctive pathophysiology, natural course, and radiographic manifestation [27]. ABL is a self-limiting remodeling process that mainly takes place in the first 6 months postoperation and will halt spontaneously after osteointegration is completed. In contrast, osteolysis involves the inflammation process, often occurring years after the operation, during which the wear debris accumulates. It may cause implant failure and necessitate revision surgery [4, 28, 29]. On plain radiographs and computed tomography, bone loss appears as a change in body contour, but the bone cortex and density are often preserved, while osteolysis manifests as osteolytic cystic lesions with disruption of the bone cortex (Figures 7 and 8). The differences in time course and radiographic characteristics between bone loss and osteolysis mean that they are distinguishable from one another at any stage.

### 4.6. Hybrid Surgery Was Associated with Less ABL after CDA with Baguera C Discs

Hybrid surgery, i.e., concomitant anterior cervical discectomy and fusion with CDA, was associated with a lower incidence of ABL, probably due to diminished micromotion, compared to CDA alone. These results were consistent with those from a similar study of Prestige-LP CDA [13], but different from those of another study of CDA with Bryan Discs [9]. In the Prestige-LP study, cervical immobilization following hybrid surgery was proposed as the reason for diminished micromotion and a lower incidence of ABL. We agree that diminished micromotion plays a major role in the difference between hybrid surgery and CDA alone. However, immobilization with a neck collar was applied for only 6 weeks after hybrid surgery in our patients, so its effect on ABL was doubtful [30]. Why ABL was not associated with hybrid surgery in the study of Bryan Discs remains unclear.

### 4.7. Limitations

There are limitations to the current study. First, there were no pain or functional outcome scores to correlate with the result of comparative radiographs and ABL. Second, because we tried to minimize the intervariability between surgeon experience, implants, techniques, and institutions, the generalizability of our findings was limited by reviewing cases operated on by the same surgeon using the same technique and the same procedure, with follow-up in a single institution. This, however, is both a weakness of our study and a strength. Third, radiological parameters were evaluated based on lateral radiographs; factors including patient position, anatomical area of coverage, and radiographic technique may have confounded our findings. Fourth, the follow-up duration was only one year; the relationship between HO and ABL, implant subsidence due to severe ABL, ABL-related adjacent disease, and reconstitution and downgrading after ABL may require further long-term follow-up. Biomechanical studies, both *in vivo* and *in vitro,* should be conducted to determine the genesis of ABL.

## 5. Conclusions

ABL is more common in Baguera C Disc arthroplasty than in Bryan Disc arthroplasty. A larger shell angle was related to ABL after CDA with Baguera C Discs, which serves as persuasive evidence that shell angle plays a pivotal role in predicting the incidence of ABL after CDA. A female predominance was found in ABL with Baguera C Disc arthroplasty, which might be related to the smaller endplate length as well as the smaller endplate-implant mismatch in females. The mismatch between the endplate and the artificial disc (or footprint mismatch) played a major role in postoperative bone homeostasis: a smaller mismatch would favor bone resorption, and a larger mismatch, or larger REE, would favor bone formation leading to HO. The association of ABL with hybrid surgery was found in CDA with Baguera C Discs, but not with Bryan Discs.

## Figures and Tables

**Figure 1:** Schematic drawings showing radiological measurements of postoperative lateral radiograms in the neutral, flexion, and extension positions.

**Figure 2:** Proposed classification of anterior bone loss by grade. Grade 0, no remodeling; grade 1a, spur disappearance without change in body contour; grade 1b, change in body contour without exposure of artificial disc; grade 2, obvious bone regression with artificial disc exposure.

**Figure 3:** Radiographic images of different grades of anterior bone loss (ABL). (a) No ABL was noted through the follow-up period (grade 0). (b) Resorption of marginal spurs was found in both the upper and lower adjacent vertebrae at 3 months postoperation. Note that there was no change in body contour, and this condition was classified as grade 1a ABL. (c) Change in body contour was found in both the upper and lower adjacent vertebrae at 6 months postoperation. These changes were classified as grade 1b ABL. (d) Grade 2 ABL was found in the upper and lower adjacent vertebrae at 3 months postoperation. (e) Resorption of anterior marginal spurs over the upper and lower adjacent vertebrae at 1.5 months postoperation was considered grade 1a ABL. The ABL progressed by 6 months postoperation to a change in body contour (grade 1b). (f) Grade 1 ABL was noted at 6 months postoperation over C5. At 12 months postoperation, the ABL at C5 progressed to grade 2. Grade 1 ABL over C6 was also noted at 12 months postoperation.

**Figure 4:** Postoperative bone loss over 12 months. Peak anterior bone loss of both the upper (a) and lower (b) adjacent vertebrae occurred within the first 6-12 months after cervical disc arthroplasty.

**Figure 5:** The key difference between Baguera C Discs and Bryan Discs. Bryan Discs have perpendicular, punched flanges which prevent posterior displacement of the device into the spinal canal. In contrast, Baguera C Discs are placed deeper, with the posterior aspect of the shell parallel to the posterior aspect of the vertebral body. Also, note the evenly distributed loading force in the neutral position.

**Figure 6:** Schematic drawings of artificial discs during flexion (a, b) and extension (c, d) for the Baguera C Discs (a, c) and Bryan Discs (b, d). The larger shell angle results in less loading force in the anterior aspect, leading to anterior bone loss, regardless of implant type.

**Figure 7:** Sample patient showing anterior bone loss (ABL). (a) Lateral radiograph of a 45-year-old woman taken one month after cervical disc arthroplasty with Bryan Disc over the C4-C5 level. (b, c) Computed tomography scan of the same patient 8 years postoperation found grade 2 ABL. Note the preserved cortex and bone density.

**Figure 8:** Sample patient showing osteolysis. (a) Lateral radiograph of a 45-year-old man taken two months after cervical disc arthroplasty with Bryan Discs over the C4-C5 and C5-C6 levels. (b, c) Computed tomography scan of the same patient 5 years postoperation found osteolysis over the posterior aspect of the C4 body.

**Table 1:** The demographic and clinical features of 77 patients receiving Baguera C Disc arthroplasty.

Characteristics	Value
Mean age, years	55.9
Sex	
Female	40
Male	37
Operative segments	
C3-C4	17 (22.0%)
C4-C5	20 (26.0%)
C5-C6	37 (48.0%)
C6-C7	3 (4.0%)
Hybrid surgery	39 (50.6%)
Anterior bone loss (%)	
Upper level (grade 1 and grade 2)	56 (72.7%)
Lower level (grade 1 and grade 2)	52 (67.5%)
Both upper and lower level	49 (63.6%)
Either upper or lower level	59 (76.6%)

**Table 2:** Anterior bone loss of the upper adjacent level by grade.

	Grade 0 and grade 1 (*n* = 57)		Grade 2 (*n* = 20)		*p* value
Sex					0.001^∗∗^
Female	23	(40.4%)	17	(85.0%)	
Male	34	(59.6%)	3	(15.0%)	
Age, years	57.0	(50.0, 65.0)	54.0	(43.5, 63.8)	0.260
Operative level					0.312
C3-C4	14	(24.6%)	3	(15.0%)	
C4-C5	17	(29.8%)	3	(15.0%)	
C5-C6	24	(42.1%)	13	(65.0%)	
C6-C7	2	(3.5%)	1	(5.0%)	
Hybrid					0.016^∗^
No	23	(40.4%)	15	(75.0%)	
Yes	34	(59.6%)	5	(25.0%)	
Depth of Baguera C Disc (mm)					0.037^∗^
13	0	(0.0%)	1	(5.0%)	
14	16	(28.1%)	10	(50.0%)	
16	41	(71.9%)	9	(45.0%)	
Height of Baguera C Disc (mm)					0.001^∗∗^
5	10	(17.5%)	12	(60.0%)	
6	43	(75.4%)	8	(40.0%)	
7	4	(7.0%)	0	(0.0%)	
Adjusted preoperative disc height (mm)	4.71	(3.78, 5.49)	3.95	(3.61, 4.78)	0.017^∗^
Postoperative measurements					
Global alignment angle	19.0	(10.5, 26.0)	17.5	(10.0, 24.0)	0.688
Lordotic angle	6.0	(2.0, 13.0)	7.5	(3.5, 13.8)	0.222
Shell angle	0.0	(-3.0, 3.5)	2.0	(-0.8, 6.8)	0.042^∗^
Global ROM	43.0	(32.5, 52.5)	52.0	(29.3, 64.0)	0.205
Index level ROM	14.0	(10.0, 20.0)	17.0	(12.3, 24.8)	0.207
Adjusted anteroposterior diameter of the upper adjacent endplate (mm)	18.4	(17.4, 19.1)	16.3	(15.8, 17.1)	<0.001^∗∗^
Mismatch (difference) between the implant and the upper adjacent endplate (mm)	2.7	(2.1, 3.3)	1.7	(1.1, 2.3)	0.001^∗∗^

Chi-square test. Mann–Whitney *U* test, median (interquartile range). ^∗^*p* < 0.05; ^∗∗^*p* < 0.01; ROM: range of motion.

**Table 3:** Anterior bone loss of the lower adjacent level by grade.

	Grade 0 and grade 1 (*n* = 65)		Grade 2 (*n* = 12)		*p* value
Sex					0.040^∗^
Female	30	(46.2%)	10	(83.3%)	
Male	35	(53.8%)	2	(16.7%)	
Age, years	56.0	(48.0, 65.0)	56.0	(46.0, 63.8)	0.983
Operative level					0.891
C3-C4	14	(21.5%)	3	(25.0%)	
C4-C5	17	(26.2%)	3	(25.0%)	
C5-C6	31	(47.7%)	6	(50.0%)	
C6-C7	3	(4.6%)	0	(0.0%)	
Hybrid					0.025^∗^
No	28	(43.1%)	10	(83.3%)	
Yes	37	(56.9%)	2	(16.7%)	
Depth of Baguera C Disc (mm)					0.410
13	1	(1.5%)	0	(0.0%)	
14	20	(30.8%)	6	(50.0%)	
16	44	(67.7%)	6	(50.0%)	
Height of Baguera C Disc (mm)					0.006^∗∗^
5	14	(21.5%)	8	(66.7%)	
6	47	(72.3%)	4	(33.3%)	
7	4	(6.2%)	0	(0.0%)	
Adjusted preoperative disc height (mm)	4.59	(3.74, 5.37)	4.05	(3.69, 5.01)	0.448
Postoperative measurements					
Global alignment angle	19.0	(10.0, 25.5)	16.5	(13.3, 24.8)	0.833
Lordotic angle	6.0	(2.0, 12.5)	7.5	(3.3, 19.8)	0.208
Shell angle	0.0	(-3.0, 4.0)	3.5	(-0.5, 6.8)	0.029^∗^
Global ROM	45.0	(33.0, 54.0)	43.0	(28.0, 55.5)	0.391
Index level ROM	15.0	(10.0, 21.5)	15.5	(11.3, 23.3)	0.725
Adjusted anteroposterior diameter of the lower adjacent endplate (mm)	17.2	(16.1, 18.5)	15.6	(14.7, 16.8)	0.002^∗∗^
Mismatch (difference) between the implant and the lower adjacent endplate (mm)	1.7	(1.1, 3.0)	0.7	(0.3, 0.9)	0.001^∗∗^

Chi-square test. Mann–Whitney *U* test, median (interquartile range). ^∗^*p* < 0.05; ^∗∗^*p* < 0.01. ROM: range of motion.

**Table 4:** Difference in adjusted anteroposterior endplate diameter by gender.

	Female (*n* = 40)		Male (*n* = 37)		*p* value
Adjusted anteroposterior diameter of the upper adjacent endplate (mm)	16.9	(16.0, 17.8)	18.8	(18.3, 20.0)	<0.001^∗∗^
Adjusted anteroposterior diameter of the lower adjacent endplate (mm)	16.2	(15.1, 17.1)	18.0	(17.1, 19.2)	<0.001^∗∗^
Mismatch (difference) between the implant and the upper adjacent endplate (mm)	2.0	(1.5, 2.8)	2.9	(2.3, 4.2)	<0.001^∗∗^
Mismatch (difference) between the implant and the lower adjacent endplate (mm)	1.1	(0.5, 1.9)	2.1	(1.1, 3.3)	0.004^∗∗^

Mann–Whitney *U* test, median (IQR). ^∗^*p* < 0.05. ^∗∗^*p* < 0.01.

## Data Availability

All data generated or analyzed during this study are included in this article. Further enquiries can be directed to the corresponding author.

## Abbreviations

ABL: Anterior bone loss
CDA: Cervical disc arthroplasty
FSU: Functional spinal unit
HO: Heterotopic ossification
REE: Residual exposed endplate
ROM: Range of motion.
